This article has been retracted.

# Deconstruction of Clinical Treatment of Pneumonia and Respiratory Tract Infection Based on MRI Molecular Imaging

**DOI:** 10.1155/2022/7146978

**Published:** 2022-09-26

**Authors:** Lili Jiang, Yan Shen, Zequan Yu, Wanli Xu

**Affiliations:** ^1^Internal Medicine, Wuhan Eighth Hospital, Wuhan 430010, Hubei, China; ^2^Department of Radiology, Wuhan Eighth Hospital, Wuhan 430010, Hubei, China

## Abstract

Pneumonia is a major research core topic in the medical field, and clinical trials of pneumonia and respiratory tract infection have been ongoing. The purpose of this study was to investigate the clinical efficacy and safety of Shuanghuanghua granules in the treatment of pneumonia and respiratory tract infection based on NMR molecular imaging, and to lay a foundation for the development of new drugs. In this paper, 126 patients were randomly divided into the control group, the treatment group 1, the and treatment group 2, and were given Fengreganmao granules, Shuanghuanghua granules (ultrafine preparation), and Shuanghuanghua granules (extract preparation), respectively. The main symptom scores, sign scores, antipyretic time, and virus content before and after treatment were recorded. Statistical analysis was carried out on this basis. The experiment showed that the body temperature of the subjects in the three groups before treatment was: control group (37.59 ± 0.78), treatment group 1 (37.8 ± 0.81), and treatment group 2 (37.6 ± 0.76). After treatment, the body temperature of subjects in the three groups was: control group (36.67 ± 0.71), treatment group 1 (36.49 ± 0.43), and treatment group 2 (36.19 ± 0.25). Experiments show that Shuanghuanghua granules can significantly reduce the nasal virus, adenovirus, parainfluenza virus, etc. in the patient's body. And it can shorten the antipyretic time of patients and has good clinical application. In addition, this study gave full play to the role of MRI molecular imaging and provided ideas and references for the clinical treatment of pneumonia and respiratory tract infection.

## 1. Introduction

Typically, acute upper respiratory tract infections have a short duration and a good prognosis. The disease has no age, no gender, no occupation, no region, and can occur throughout the year, but it is more common in winter and spring. However, it is also possible to cause widespread epidemics and even serious complications in sudden climate change, so effective preventive measures should be taken. At present, there are no specific drugs for many viral diseases, and viral diseases that can be used for prevention are rare. Moreover, due to the mutation of the virus, the clinical effect of some vaccines is greatly reduced. Moreover, most of the antiviral drugs have serious side effects, and long-term use can easily lead to drug resistance, thus affecting the efficacy. In recent years, Chinese medicine has made great progress in the treatment of viral diseases, and its antiviral effect is unmatched by other chemical drugs. For example: good efficacy, broad antiviral spectrum, low toxicity and side effects, no teratogenicity, and resistance to drug resistance. Therefore, the development of new antiviral drugs has become a research hotspot, and traditional Chinese medicine is currently a hotspot in the world.

Research on the clinical treatment of pneumonia and respiratory tract infection has been ongoing. Borgnolo determined whether antibiotic prophylaxis reduces respiratory infections and overall mortality in unselected critically ill adult patients [1]. Wieland et al. compared the agreement between standardized ultrasonography and clinical examination in the diagnosis of umbilical infection [2]. Mahashur discussed the management of clarithromycin in mild to moderate lower respiratory tract infections [3]. Juhsz et al. reviewed the clinical microbiological characteristics of bacteria, especially their role in lower respiratory tract infections and antibiotic treatment selection [4]. Karampeli et al. understood the epidemiological and clinical characteristics of patients with interstitial pneumonia with autoimmune features and observed disease progression, treatment response, and infection frequency during a 1-year follow-up period [5]. Gugu et al. identified the combined effect of snail mucin as a natural product antibacterial agent of animal origin and lincomycin against different strains of *Streptococcus pneumoniae* [6]. These studies do not allow visual inspection of the infection, so they require the assistance of molecular magnetic resonance imaging.

NMR molecular imaging has been studied by many scholars, and Konopka et al. used NMR to chemically evaluate 64Cu-Rho-G4-CML and its nontargeted analogs [7]. Mahdiyeh used radionuclide-based imaging methods for early diagnosis and treatment of cancer [8]. These studies did not carry out clinical experiments, at the same time, there is a lack of data support, so this paper studies the clinical treatment of pneumonia and respiratory tract infection based on MRI molecular imaging.

In this paper, patients in a certain hospital were taken as the research objects, and body temperature, detoxification time, peripheral blood leukocytes, and neutrophils were used as experimental indicators to observe the changes of experimental indicators in the control group, treatment group 1, and treatment group 2. The experimental results showed that the antipyretic time of the control group was 23.45 ± 12.98, the antipyretic time of the treatment group 1 was 18.49 ± 13.45, and the antipyretic time of the treatment group 2 was 13.94 ± 7.49, indicating that Shuanghuanghua granules had better antipyretic effect.

## 2. Clinical Treatment of Pneumonia and Respiratory Tract Infection

In simple terms, MRI is Fourier transformed by hardware, so by scanning the patient's body, the corresponding frequency domain information can be obtained. Although MRI has been used increasingly clinically, its slow scanning speed is an important factor restricting its application. Its slow scanning speed can cause motion artifacts and increase the difficulty of dynamic imaging. Obtaining high-resolution medical images requires more MRI technology, so how to improve the imaging speed of images under the premise of ensuring image quality is an important topic at present [9, 10].

The imaging speed of the current MRI is limited by the scanning time. The scanning time is too long for the patient to bear, and during the scanning, the patient must be completely still, which increases the difficulty of real-time imaging. The current commonly used method is to use the phased array coil to receive the induction signal and to encode the spatial position information, which greatly shortens the scanning time and speeds up the imaging speed. However, it cannot be too large, because of the limitation of spatial information, if the data is too small, the reconstructed image will produce large artifacts. Second, small samples are processed mathematically to improve the quality of the images [11, 12].

MRI is mainly composed of three basic components, namely, the magnet part, the magnetic resonance spectrometer part, the data processing part, and the image reconstruction part. The basic building blocks of MRI are shown in Figure 1 [13, 14].

The principle of MRI: the hydrogen nucleus is the most ideal human imaging nucleus [15, 16]. The intensity of the NMR signal depends on the concentration of hydrogen nuclei in the sample. Due to the different water content in the human body, that is, the number of hydrogen nuclei, the intensity of the NMR signal will also vary greatly. Under the action of the high-frequency pulse, the state of the hydrogen nuclei will change, and after the frequency, the hydrogen nuclei will return to their original energy state. Through further computer processing, the chemical composition of the reaction tissue can be obtained, to obtain the water changes and the movement of water molecules inside the tissue. In this way, pathological changes can be recorded [17, 18]. The images displayed by MRI are clear and detailed, which can greatly improve the physician's diagnosis, and can save surgical operations such as laparotomy and laparotomy. MRI is not harmful to the body because it does not generate X-rays and does not cause harm to the body [19, 20].

Pneumonia is an inflammation caused by lung tissue, lung parenchyma, and lung interstitium. The respiratory tract is the respiratory system of the human body, consisting of the upper airway and the lower airway, and the upper airway is the nasal cavity, the pharynx, and the throat, such as the upper respiratory tract, and can also be rhinitis, sinusitis, and pharyngitis. Lower respiratory tract infection mainly refers to bronchitis, that is, inflammation of the main bronchus and various sub-bronchioles. The symptoms of pneumonia are much more severe than those of a respiratory infection.

There are many ways to treat lung infection, depending on the patient's condition and cause. If it is a bacterial infection, people can take oral antibiotics, intravenous infusion, etc., and generally recover completely within half a month. If it is caused by other infections, it generally needs to be treated with antituberculosis drugs, and it can be fully recovered in about one year.

Pulmonary infection is a relatively common respiratory tract infection with symptoms in both adults and children. The treatment of pulmonary infection is mainly based on anti-infection, supplemented by corresponding treatment and supportive care. Here are five common treatments for lung infections.

1. Remove primary lesions. If the patient has inhalation injury or severe facial and neck burns, it is necessary to strengthen the management of the airway to clear the secretions and necrotic mucosa of the airway, thereby speeding up the recovery of the airway. When blood-borne pneumonia occurs, sepsis must be controlled and removed.
2. Intravenous injection. The patient's sputum culture and environment are checked for bacteria, and then intravenous injections are given.
3. Respiratory dysfunction. If combined with respiratory insufficiency, the treatment of respiratory insufficiency can be used.
4. Antibiotic treatment. If there is a *Streptococcus pneumoniae* infection, penicillins such as ceftriaxone and cefotaxime can be taken orally. For the infection of atypical pathogens, roxithromycin and ofloxacin can be selected, and macrolides and quinolones can be selected.
5. Actively cooperate with treatment. During the treatment, it is necessary to cooperate with the doctor's treatment, to take regular rest, and to quit smoking and drinking.

Lung infections are caused by various bacteria and fungi, and the length of its cure and treatment is related to the severity of the infection. If there is a lung infection, treat it under the guidance of a doctor to ensure the safety of your own life. When treating, we should pay attention to the timely discharge of sputum, mainly including spray inhalation, back path, and phlegm-reducing drugs.

Parainfluenza viruses can be divided into types 1, 2, and 3. The distribution of PIV in different regions has obvious seasonality. PIV-3 is the most prevalent disease, with outbreaks usually occurring between April and June. The incidence of PIV-1 and PIV-2 was mainly in autumn. PIV-3 is the most common pneumonia in hospitalized adults. There are several risk factors for PIV infection to develop into pneumonia and severe diseases, including older age, steroid use, and immunodeficiency. In patients with hematological malignancies and hematopoietic stem cell transplantation combined with PIV, the incidence of pneumonia was 37%. The main factors for the occurrence of lower respiratory tract infection are early infection, hormone therapy, and other pathogenic infections. A systematic review showed that in PIV pneumonia, there is an average mortality rate of 27%. Other risk factors include hormone use, infection with other pathogens, cancer recurrence, or difficulty in treatment. Most researchers focus on developing short-term intervening RNAs that target viral genes.

Adenovirus damage to the respiratory tract is often mild and limited. However, severe pneumonia, respiratory failure, and dead disease can occur in the military, some facilities, community outbreaks, or even global outbreaks. Severe adenovirus infection also occurs in hematopoietic stem cell transplant and solid organ transplant patients, which may be asymptomatic or a form of fatal pneumonia in systemic disease. After being infected with adenovirus pneumonia, the mortality rate is high. Even for patients with normal immune system, the fatality rate is as high as 26.7%, and some studies have reached 50%. In in vitro experiments, cidofovir has a good inhibitory effect on various adenovirus subtypes. A few cases reported that cidofovir with or without intravenous immune globulin in the treatment of severe adenovirus pneumonia can improve the clinical prognosis of patients, but its clinical use is limited due to its adverse reactions and adverse reactions. The combination of hydration and benecid can prevent kidney damage. Brincidofovir (CMX001) is a cidofovir lipid-binding agent with good oral absorption, which has good application prospects.

Viral pneumonia and bacterial pneumonia are two different types of pneumonia, and the treatment methods of the two are also very different. Viral pneumonia is an inflammation of the lungs that can be transmitted to the lungs by a virus in the upper respiratory tract. Viral pneumonia can appear throughout the season, but is more common in winter and spring. Viral pneumonia can break out, or it can spread. It is mainly due to inhalation infection, or mainly due to the transmission of droplets, and generally manifests as fever, headache, cough, and a small amount of white mucus. The virus slowly invades the upper respiratory tract, damages the upper respiratory tract, weakens its immunity, and eventually causes bacterial infection. If not dealt with in time, a large number of bacteria and viruses will slowly spread, eventually resulting in interstitial pneumonia. Treatment should pay more attention to rest, pay more attention to maintaining indoor air circulation, and open more windows. At the same time, it is necessary to strengthen the isolation to prevent cross-infection. Some common diseases, such as influenza and parainfluenza, are caused by a large number of bacteria and viruses, resulting in viral pneumonia. *Streptococcus pneumoniae*, *Haemophilus* influenzae, and *Staphylococcus aureus* are the most common pneumoniae. These symptoms can vary widely, from mild to severe, mainly because of the pathogen and host conditions. The symptoms include cough, expectoration, or exacerbation of original respiratory symptoms, purulent or bloody sputum, with or without chest pain. The treatment of bacterial pneumonia is mainly antibiotics. If you cough a lot, you need to use drugs for cough and phlegm The treatment of viral pneumonia is mainly antivirus, heat-clearing, and detoxification. Bacterial pneumonia is generally caused by *Streptococcus pneumoniae* or other common bacterial infections, with clinical manifestations such as fever, cough, and expectoration.

The causative microorganisms of upper respiratory tract infection account for 70% to 80%, the causative microorganism of lower respiratory tract infection accounts for 6% to 61%, and among the causative microorganisms of community-acquired pneumonia, 2% to 30% are viruses. In recent years, the detection rate of viral pneumonia has increased significantly. About 22% of viral pneumonia cases in US. hospitals are viral, while bacterial pneumonia accounts for only 11%, and viral pneumonia is only 3%. In addition, influenza outbreaks have concentrated short-term outbreaks and seasonal epidemics in various regions, and many variants have emerged. Because the human body is highly sensitive to viruses that cause respiratory infections, and the virus has strong intracellular parasiticity, it is prone to mutation and drug resistance, which brings certain difficulties to clinical diagnosis and treatment. The treatment of respiratory tract infection is mainly in the emergency department, and there is an urgent need for timely, standardized, and accurate diagnosis and rational application of antiviral drugs.

In vitro isolation and culture is the current standard for viral etiology diagnosis, but this technology is not only time-consuming and has a low positive rate, but also some clinically relevant viruses (such as rhinovirus, coronavirus) are difficult to grow in traditional culture methods. Therefore, the application in in vitro isolation and culture is limited. Antibodies usually appear 1–2 weeks after virus infection, and serum detection sensitivity is low and cannot be detected in time. At present, the commonly used antigen detection methods are: ELISA, colloidal gold immunoassay, immunochromatography, etc., but the detection of antigen must collect a sufficient number of cells, generally from nasopharyngeal, tracheal aspirates, and bronchoalveolar lavage fluid. Because the number of cells obtained from the throat swabs is low, there is a certain error in antigen detection. As a fast, simple, and automated pathogenic detection technology, point-of-care detection has great differences in detection range, detection technology, detection range, and sensitivity of kits, which will have a certain impact on the detection results. It was reported that a single-tube multiplex PCR technique was used to detect 22 pathogenic bacteria associated with respiratory tract infections at one time. The sensitivity of PCR detection of respiratory viruses is 2 to 5 times that of traditional virus antibody, antigen, and culture detection methods. Especially in the case of adults and the elderly with low virus content in the nasopharynx, PCR detection has obvious advantages. In a randomized controlled trial, patients who underwent POCT with PCR had a shorter mean hospital stay (5.7 days) than the control group (6.8 days). Another multicenter randomized controlled study showed that the median antiviral duration of PCRPOCT patients was 1 hour, which was significantly lower than that of the control group at 6 hours, and the incidence of adverse reactions in the POCT group was also lower. Next-generation metagenomic sequencing (mNGS) can analyze the genome structure of all microorganisms including bacteria, viruses, and fungi on the basis of one-time sequencing, thereby helping people to quickly identify pathogenic bacteria.

Most viruses can be detected within 2 days of onset, and the number of viruses in respiratory samples will gradually decrease over time, as a result, the number of viruses is too small, resulting in erroneous results. When rhinovirus infection occurs, the peak of nucleic acid amplification is 2 days after the onset of the disease, and the number of viruses will drop rapidly after up to 7 days. The peak of metapneumovirus nucleic acid amplification in 57% of the people occurred 2 days after the onset of the disease, and only 19% of the people had an increase in the number of metapneumoviruses 4 days after the onset of the disease. While four days after the onset of symptoms, only 27% were positive. In the detection of upper respiratory syncytial virus in children, it was found that within 2 days after infection, the virus continued to fall off for 4.5 days, and the best time for influenza virus was 1 day after the onset, and the longest was 6 to 8 days. Bacterial or fungal infection secondary to acute respiratory viral infection in adults is relatively rare, mainly caused by respiratory bacterial infection, and bacterial pneumonia is very different from pure respiratory viral infection (or viral pneumonia). Bacterial pneumonia occurs in 15% of pneumonia patients, mainly caused by rhinovirus and streptococcal infections. Current studies have shown that among mixed infections, *Streptococcus pneumoniae*, *Haemophilus* influenzae, and *Chlamydia pneumoniae* are the most common, followed by rhinovirus, influenza A virus, and adenovirus. Different studies have shown that co-infections cause more clinical symptoms and complications, including body temperature, length of hospital stay, and risk of death, but there were no significant differences in CURB-65 and PSI scores.

The laboratory diagnosis methods of respiratory virus infection mainly include four types: virus isolation and culture, antigen detection, serum immunological antibody detection, and nucleic acid detection. Laboratory diagnostic methods for respiratory viral infections are shown in Figure 2.

In this paper, the clinical treatment of pneumonia and respiratory tract infection was studied by using nuclear magnetic resonance molecular imaging technology. For the one-dimensional signal *ε*, the sensing matrix *γ* of *α∗β* (*α* ≪ *β*) was used to lose characteristic information, then:

(1) $$\begin{array}{c} \delta =\gamma \varepsilon \text{.} \end{array}$$

Let {*η*_*ζ*_}_*ζ*=1_^*β*^ be an orthogonal base composed of *β∗*1 column vectors, and *θ* be an orthogonal matrix of *β∗β*, then the signal has a sparse representation with a sparsity of *ι*:

(2) $$\begin{array}{c} \varepsilon \approx \sum_{\zeta =1}^{\iota }\kappa_{\zeta }\eta_{\zeta }\text{.} \end{array}$$

And:

(3) $$\begin{array}{c} \varepsilon =\eta \kappa \text{.} \end{array}$$

Then:

(4) $$\begin{array}{c} \delta =\gamma \eta \kappa \text{.} \end{array}$$

Sparse optimization problem model:

(5) $$\begin{array}{c} \min{\left\|\kappa \right\|}_{0}\;s.t.\delta =\lambda \kappa \text{.} \end{array}$$

Among them, *λ*=*γη*.

Use the norm instead:

(6) $$\begin{array}{c} \min{\left\|\kappa \right\|}_{1}\;s.t.\delta =\lambda \kappa \text{.} \end{array}$$

This problem is a convex optimization problem.

Mathematical model of MRI:

(7) $$\begin{array}{c} \min{\left\|\mu \alpha \right\|}_{0}\;s.t.{\left\|\nu \alpha -\delta \right\|}_{2}<\xi \text{.} \end{array}$$

Among them, *μ* represents the sparse transform, *ν* represents the partial Fourier transform, and *ξ* represents the allowable error vector.

The imaging model for reconstructing the MRI image from the sampled data *ϖ* is as follows:

(8) $$\begin{array}{c} \min{\left\|\eta \varepsilon \right\|}_{1}\;s.t.{\left\|\varpi -\nu \varepsilon \right\|}_{2}\leq \xi \text{.} \end{array}$$

Imaging model based on local sparse dictionary:

(9) $$\begin{array}{c} \min\left\{{\left\|\rho \varrho -\sigma \right\|}_{1}\right\}s.t.{\left\|\nu \right\|}_{2}\leq \varsigma \text{.} \end{array}$$

Among them, *ρ* is image patch extraction operations, *ϱ* is local sparse dictionaries, and *σ* is sparse levels.

Objective function:

(10) $$\begin{array}{c} \min\left\{{\left\|\tau \right\|}_{1}+\sum \varrho \sigma \right\}s.t.{\left\|\varsigma \right\|}_{2}\leq \varphi \text{.} \end{array}$$

Locally sparse:

(11) $$\begin{array}{c} \min\;\sum \varrho \sigma \;s.t.{\left\|\varsigma \right\|}_{2}\leq \varphi \text{.} \end{array}$$

Rebuild the subproblem:

(12) $$\begin{array}{c} \min\;\phi \left(\varepsilon \right)={\left\|\nu \alpha -\delta \right\|}_{2}^{2}+\sum {\left(\rho \varrho -\sigma \right)}^{2}\text{.} \end{array}$$

Gradient of *ϕ*(*ε*):

(13) $$\begin{array}{c} ⋁\phi \left(\varepsilon \right)=2\tau \sum \varsigma \tau +{\left(\rho \varrho -\sigma \right)}^{2}\text{.} \end{array}$$

It can be further optimized:

(14) $$\begin{array}{c} ⋁\phi \left(\varepsilon \right)=2\tau \left[{\varsigma \tau +\left(\rho \varrho -\sigma \right)}^{2}\right]\text{.} \end{array}$$

Intermediate image:

(15) $$\begin{array}{c} \tau =\frac{\sum \upsilon^{T}\tau_{\zeta }}{\omega }\text{,}\\ \omega =\frac{\Gamma }{\Theta^{2}}\text{.} \end{array}$$

Among them, Γ is the number of pixels in the image block, and Θ is the overlap distance between two adjacent image blocks.

## 3. Therapeutic Effect

All patients with acute upper respiratory tract infection were treated or emergency patients who visited the Affiliated Hospital of the Chinese Academy of Medical Sciences between October 2021 and April 2022, and the course of the disease was within 24 hours.

The included subjects were randomly divided into three groups: treatment group 1, treatment group 2, and control group according to the ratio of 1 : 1:1, with 42 cases in each group. SAS software was used to generate random numbers to determine the coding of the three groups of drugs, and the drugs were coded blind according to the requirements of double-blind clinical trials. The blinding process has detailed blinding records for future reference, and the blinded drug codes are sealed and handed over to clinical researchers for preservation. Only in the event of an emergency for the subject, the blinding can be broken urgently.

### 3.1. Control Group

Shuanghuanghua granule No. 1 (Fengregan granules group); Treatment group 1: Shuanghuanghua granule No. 2 (Shuanghuanghua granules, ultrafine preparation group). Treatment group 2: Shuanghuanghua granule No. 3 (Shuanghuanghua granule extraction preparation group). The three groups were all taken with boiled water, 1 bag at a time, 3 times a day, and the course of treatment was 3 days.

The rank sum test, also known as the order sum test, is a nonparametric test. It does not depend on the specific form of the overall distribution and can be applied regardless of the distribution of the object to be studied and whether the distribution is known, so it is highly practical. The comprehensive efficacy evaluation of disease and syndrome compiled a frequency table in frequency format, the overall efficacy and total effective rate of each group were calculated, and the rank sum test was used to compare between groups. The main symptoms of the subjects were described as the mean ± standard deviation (M ± SD) to describe the disappearance time. And the frequency table was used to describe the changes before and after treatment, the scores before and after treatment were analyzed by rank sum test, and the differences within and between groups were analyzed by *t*.

The gender distribution of the subjects is shown in Table 1.

Table 1 shows that the number of subjects in the three groups is 42. Among them, the control group (male: 21, female: 21), treatment group 1 (male: 23, female: 19), and treatment group 2 (male: 22, female: 20).

The age comparison results of the subjects are shown in Table 2.

Table 2 shows that the ages of the three groups of subjects are: the control group (25.67 ± 6.23), the treatment group 1 (25.89 ± 5.75), and the treatment group 2 (26.38 ± 6.43). The minimum age of the subjects in the three groups is 18 years old. It can be clearly seen that there is no significant difference in the age of the three groups of subjects.

The results of the height comparison of the subjects are shown in Table 3.

Table 3 shows that the heights of the three groups of subjects are: control group (164.95 ± 7.12), treatment group 1 (166.12 ± 6.83), and treatment group 2 (165.46 ± 7.47). It can be clearly seen that there is no significant difference in the height of the three groups of subjects.

The weight comparison results of the subjects are shown in Table 4.

Table 4 shows that the body weights of the three groups of subjects are: the control group (63.17 ± 6.13), the treatment group 1 (62.48 ± 5.79), the treatment group 2 (61.93 ± 5.56). It can be clearly seen that there is no significant difference in the body weight of the three groups of subjects.

The results of the disease efficacy comparison of the subjects are shown in Table 5.

Table 5 shows the total effective rate of the three groups of diseases: control group (71.43%), treatment group 1 (88.10%), treatment group 2 (88.10%), and the ineffective rates were 28.57%, 11.90%, and 11.90%, respectively.

The results of the comparison of the efficacy of the syndromes of the subjects are shown in Table 6.

Table 6 shows the total effective rate of the three groups of syndromes: control group (71.43%), treatment group 1 (90.47%), treatment group 2 (85.71%), and the ineffective rates were 28.57%, 9.53%, and 14.29%, respectively.

The comparison results of the subjects' body temperature before and after treatment are shown in Figure 3.

Figure 3 shows that the body temperature of the subjects in the three groups before treatment is: control group (37.59 ± 0.78), treatment group 1 (37.8 ± 0.81), and treatment group 2 (37.6 ± 0.76). After treatment, the body temperature of the subjects in the three groups was: control group (36.67 ± 0.71), treatment group 1 (36.49 ± 0.43), and treatment group 2 (36.19 ± 0.25). There was no significant difference in the results of the treatment group 1 and the treatment group 2 compared with the control group.

The comparison results of the subjects' antipyretic time before and after treatment are shown in Figure 4.

Figure 4 shows that the antipyretic time of the control group was 23.45 ± 12.98, the antipyretic time of the treatment group 1 was 18.49 ± 13.45, the antipyretic time of the treatment group 2 was 13.94 ± 7.49. There were significant differences in the results of the treatment group 1 and the treatment group 2 compared with the control group.

The comparison results of the subjects' peripheral blood leukocytes before and after treatment are shown in Figure 5.

Figure 5 shows the peripheral blood leukocyte content of the three groups before treatment: control group (4.48 ± 0.48), treatment group 1 (4.53 ± 0.62), and treatment group 2 (4.46 ± 0.33). After treatment, the peripheral blood leukocyte content in the three groups was: control group (4.58 ± 0.44), treatment group 1 (4.74 ± 0.81), and treatment group 2 (4.72 ± 0.36). There was no significant difference in the results of the treatment group 1 the and treatment group 2 compared with the control group.

The comparison results of the subjects before and after treatment with peripheral neutrophils are shown in Figure 6.

Figure 6 shows the levels of peripheral neutrophils in the three groups before treatment: control group (3.45 ± 0.82), treatment group 1 (3.13 ± 0.87), and treatment group 2 (4.82 ± 1.42). After treatment, the peripheral neutrophil content of the three groups of subjects was: control group (3.59 ± 0.53), treatment group 1 (3.52 ± 0.8), and treatment group 2 (4.51 ± 1.14). There was no significant difference in the results of the treatment group 1 and the treatment group 2 compared with the control group.

## 4. Conclusions

To test the clinical therapeutic effect of Shuanghuanghua granules on pneumonia, and respiratory tract infection, three groups of treatment plans were designed by using nuclear magnetic resonance molecular imaging technology in this study, namely, the control group, the treatment group 1, and the treatment group 2. The results of this experiment show that the three groups of treatment methods can effectively control wind-heat obstruction lung combined with Qi deficiency syndrome, the total effective rates are 71.43%, 88.10%, and 88.10%, the ineffective rates are 28.57%, 11.90%, and 11.90%. Shuanghuanghua granule has a significant effect on the treatment of acute upper respiratory tract infection with wind-heat obstruction and qi deficiency syndrome. It can not only significantly improve its clinical symptoms, but also significantly reduce rhinovirus, adenovirus, and parainfluenza virus in serum, and at the same time shorten the antipyretic time of fever patients. To further verify the antipyretic and antiviral effects of Shuanghuanghua granules, it is necessary to expand the scope of investigation, increase the number of hospitals under investigation, and adopt better laboratory methods such as molecular biology, proteomics, and serum pharmacology, to better understand the relationship between drugs and viruses, to better guide clinical work, give full play to the advantages of traditional Chinese medicine, and lay a solid foundation for the development of new antirespiratory virus drugs.

## Figures and Tables

**Figure 1:** Basic building blocks of MRI.

**Figure 2:** Laboratory diagnostic methods for respiratory viral infections.

**Figure 3:** Comparison results of subjects' body temperature before and after treatment.

**Figure 4:** Comparison results of subjects' antipyretic time before and after treatment.

**Figure 5:** Comparison results of subjects' peripheral blood leukocytes before and after treatment.

**Figure 6:** Comparison of results before and after treatment with peripheral neutrophils in subjects.

**Table 1:** Gender distribution of subjects (cases).

Group	Number of examples	Male	Female
Control group	42	21	21
Treatment group 1	42	23	19
Treatment group 2	42	22	20

**Table 2:** Subject age comparison (years).

Group	M ± SD	Maximum value	Minimumvalue
Control group	25.67 ± 6.23	54	18
Treatment group 1	25.89 ± 5.75	52	18
Treatment group 2	26.38 ± 6.43	48	18

**Table 3:** Subject height comparison (cm).

Group	M ± SD	Maximum value	Minimumvalue
Control group	164.95 ± 7.12	182	156
Treatment group 1	166.12 ± 6.83	176	158
Treatment group 2	165.46 ± 7.47	179	157

**Table 4:** Subject weight comparison (kg).

Group	M ± SD	Maximum value	Minimumvalue
Control group	63.17 ± 6.13	81	45
Treatment group 1	62.48 ± 5.79	89	48
Treatment group 2	61.93 ± 5.56	86	46

**Table 5:** Comparison of disease efficacy of subjects (cases).

Group	Clinical recovery	Effective	Efficient	Invalid	Total efficiency (%)
Control group	9	11	11	12	71.43
Treatment group 1	11	17	9	5	88.10
Treatment group 2	10	19	8	5	88.10

**Table 6:** Comparison of syndrome and efficacy of subjects (example).

Group	Clinical recovery	Effective	Efficient	Invalid	Total efficiency (%)
Control group	9	10	12	12	71.43
Treatment group 1	11	17	10	4	90.47
Treatment group 2	10	19	7	6	85.71

## Data Availability

The data underlying the results presented in the study are available within the manuscript.
